# Integrated phosphorus nutrient sources improve wheat yield and phosphorus use efficiency under sub humid conditions

This article has been retracted.

**DOI:** 10.1371/journal.pone.0255043

**Published:** 2021-10-06

**Authors:** Khuram Mubeen, Allah Wasaya, Haseeb ur Rehman, Tauqeer Ahmad Yasir, Omer Farooq, Muhammad Imran, Rao Muhammad Ikram, Rabiah Nazeer, Faisal Zahoor, Muhammad Waqas Yonas, Mudassir Aziz, Muhammad Habib-ur-Rahman, Matlob Ahmad, Mahmood Alam, Muqarrab Ali, Mazhar Ali, Abdul Khaliq, Muhammad Ishtiaq, Muhammad Mohsin Waqas

**Affiliations:** 1 Department of Agronomy, MNS University of Agriculture, Multan, Pakistan; 2 College of Agriculture, Bahauddin Zakaria University, Multan, Pakistan; 3 Department of Agronomy, Bahauddin Zakaria University, Multan, Pakistan; 4 Department of Soil and Environmental Sciences, MNS University of Agriculture, Multan, Pakistan; 5 Department of Agronomy, The University of Poonch Rawalakot, Rawalakot, Azad Jammu and Kashmir, Pakistan; 6 Department of Agricultural Engineering, Ghazi University, Dera Ghazi Khan, Pakistan; 7 Department of Seed Science and Technology, MNS University of Agriculture, Multan, Pakistan; 8 Department of Environmental Sciences, COMSATS University Islamabad, Islamabad, Pakistan; 9 Soil and Water Testing Laboratory, Kotla Ahmad Road, Rajanpur, Pakistan; 10 Institute of Plant Protection, MNS University of Agriculture, Multan, Pakistan; 11 Department of Agricultural Engineering, Khwaja Fareed University of Engineering and Information Technology, Rahim Yar Khan, Pakistan; Anhui Agricultural University, CHINA

## Abstract

Majority of Pakistani soils are deficient in phosphorus. Phosphorus is usually applied in form of synthetic fertilizer. However integrated use of P from synthetic and organic sources can be more profitable and beneficial on sustainable basis. Field trials were conducted at research farm University of Poonch, Rawalakot, AJK, Pakistan for two consecutive years to check the comparative effects of synthetic fertilizer and organic manures applied alone and in combinations on the phosphorus use efficiency (PUE), wheat yield and yield components. Shafaq-06 cultivar of wheat was used as test cultivar. Ten treatments were included: (I) Control (P_0_) without application of fertilizer; (II) SSP @ 60 kg/ha (P_60SSP_); (III) SSP @ 90 kg/ha (P_90SSP_); (IV) SSP @ 120 kg/ha (P_120SSP_); (V) PM @60 kg/ha (P_60PM_); (VI) PM @90 kg/ha (P_90PM_); (VII) PM @120 kg/ha (P_120PM_); (VIII) SSP @30 kg/ha + PM @30 kg/ha (P_30SSP+30PM_); (IX) SSP @45 kg/ha + PM @45 kg/ha (P_45SSP+45PM_); (X) SSP @60 kg/ha + PM @60 kg/ha (P_60SSP+60PM_) which were laid out under the Randomized Complete Block Design. Significantly higher values for yield of grain (2397 kg/ha) was recorded with PM + SSP @ 60 kg P_2_O_5_ ha^-1^ each. Likewise, FPUE, PIR of wheat and AFPUE was quite higher with combined use of PM and SSP i.e. P_60SSP+60PM_ treatment. Additionally, increase in PUE, wheat yield and yield components associated with combined treated plot would help to minimize the use of high cost synthetic mineral fertilizers and represents an environmentally and agronomically sound management strategy.

## 1. Introduction

Wheat crop growth and yield is significantly influenced by phosphorus [1]. Early stages of wheat crop required phosphorus for proper growth and good yield of wheat crop [2]. Adequate amount of phosphorus enhances the root growth and seedling establishment of wheat crop [3]. Phosphorus as a basic nutrient plays a vital role from seedling to maturity stage of plant. Besides, all phonological, physiological and morphological processes improvement it also helps to enhance quality and as well as number of seeds on a plant [4].

So, sufficient supply of P is necessary particularly at early crop growth stage. Insufficient supply will be resulted in irreversible way, even P supply is started to apply in a sufficient amount [5]. Furthermore, phosphorus improves wheat crop tillering stage and brings uniformity at heading stage. It also increases the WUE of crop plant which ultimately increases the wheat potential of GY [6]. Synthetic fertilizer of phosphorus includes SSP, TSP, DAP, DCP etc. While organic sources include FYM (farmyard manure), PL (poultry litter), PM (poultry manure), compost and vermi-compost etc. Balanced use of fertilizer particularly NPK perform a fundamental role in enhancing yield and quality of wheat crop [7]. No doubt, inorganic sources enhances crop yield very quickly but their unwise use is very hazardous for the environment [8]. While, natural sources not just supply adequate N.P.K but also show good effect on the plant growth and development, water holding capacity (WHC), improving the fertility of the soil and also enhancing the biological characteristics of the soil [9].

Poultry manure is a cheap and excellent source of phosphorus among all organic fertilizer sources. Poultry manure is the farm fowl’s excreta which gradually decompose and contain high percentage of P as compared to any other organic nutrient sources. It contains around 3.03% nitrogen, 2.63% phosphorus and 1.4% potash [10]. Under conditions of higher fertilizer rates, shortage at planting time and insufficient availability of inorganic fertilizers source [11] crop grower may be motivated to apply low cost and readily accessible natural waste as fertilizer of phosphorus (P) and all essential macro-nutrients. This practice may enhance the N: P, organic matter of the soil, availability of the necessary micronutrient [12].

However, only organic manure application is insufficient to obtain higher yield. Organic manures are applied in larger amount to meet-up the crop requirement due to relatively less nutrient percentage [13]. Organic manure helps the crop plant in multiple ways by providing balanced nutrient. This could be due to improve in increased soil microbial activity which improves soil nutrient availability and decomposition of harmful elements [14]. That’s why combined use of synthetic and natural fertilizers enhances the fertilizer PUE and yield of crop [15]. Complementary use of inorganic and organic fertilizers is very important for increasing the FUE and decreasing the hazards produced by the unwise use of synthetic fertilizers, respectively [16].

It is commonly agreed that for assessment of high-potential new cultivar, application of higher rate of phosphorus fertilizer is pre-requisite [17]. Rice genotype with higher PUE adapted in those soils where low P availability in cultivated soils would help to improve the grains yield [18] because it encourages the root development and assist for the nitrogen uptake which ultimately enhances the protein content in the grain [19]. More effective utilization of phosphorus is required to increase the beneficial life of phosphorus in globe, for producing more food at low cost and to enhance the value of economic yield of the crop [20]. As developing countries are facing poverty and food security they are facing largely low P level in soils. Many efforts are done at global to quantify the P reserve in soil [21]. Hence, the significance of phosphorus (P) fertilizer as a major crop nutrient in this experiment was set to check relative impact of sources of phosphorus (P) fertilizer (synthetic and organic) which is used sole or in several combinations on PUE (phosphorus use efficiency) and the wheat yield under the sub humid environment.

## 2. Materials and methods

### 2.1 Site

The field study was performed at farm area of University of Poonch, Rawalakot, AJK for two consecutive growing seasons of 2011 and 2012.

### 2.2 Treatments and crop husbandry

Wheat cultivar Shafaq-06 was cultivated as a test wheat cultivar. Treatments included: (I) Control (P_0_) No application of fertilizer; (II) SSP @ 60kg/ha (P_60SSP_); (III) SSP @ 90kg/ha (P_90SSP_); (IV) SSP @ 120kg/ha (P_120SSP_); (V) PM @60 kg/ha (P_60PM_); (VI) PM @90 kg/ha (P_90PM_); (VII) PM @120 kg/ha (P_120PM_); (VIII) SSP @30 kg/ha + PM @30 kg/ha (P_30SSP+30PM_); (IX) SSP @45 kg/ha + PM @45 kg/ha (P_45SSP+45PM_); (X) SSP @60 kg/ha + PM @60 kg/ha (P_60SSP+60PM_) which were laid out under Randomized Complete Block Design having three replications. Wheat seed was used at the rate of 120 kg/ha and the sowing was done by using hand drill under rain fed sub humid conditions.

### 2.3 Soil and plant analyses

Prior to sowing, soil sample was collected and dried in the air. Pestle and mortar was used to grind the soil then screened out from 2mm sieve [22]. Nelson and Sommers’s proposed method was used to determine the total carbon and P in soil [23]. Hydrometer-method was used to check the distribution of the soil-particle size [24]. While the pH was determined by the Mclean’s method by the saturated soil solution with 1:1 proportion of soil and water [25]. Similarly, Kjeldahl method was used to extract total nitrogen content in soil [26]. Total extractable K (potassium) was measured by Richards’s procedure [27].

Alongside soil analysis, poultry-manure analysis was additionally done in the same institute’s laboratory after collecting the composite sample from the grower’s field. After drying in the air, grinding and screening through the 2mm sieve to get homogenize manure sample free from undesired particles was obtained. To determine total P in the plant hot-plate digestion strategy was practiced and absorbance of total plant P was measured by using Spectrophotometer at λ of 410 nm [28]. While phosphorus (P) % in plants body was determined according to following formula:

$$\text{Phosphorus}\;\%\;\text{in}\;\text{plant}=\frac{\text{Total}\;\text{phosphorus}\;\text{in}\;\text{plant}\times \text{Volume}\;\text{of}\;\text{Digest}}{\text{Total}\;\text{weight}\;\text{of}\;\text{crop}\times 1000}$$

### 2.4 Observations

Observations of wheat plant on Leaf area (cm^2^), Leaf moisture content (%), PH (PH cm), spike length (SL cm), no. of grains (spike^-1^), 1000-grain weight (TGW g) and GY (GY k/ha) were recorded. While FPUE (fertilizer phosphorus use efficiency), AFPUE (applied fertilizer phosphorus uptake efficiency) and Phosphorus-index ratio (PIR) were measured according to the following formulae [29].

$$\text{FPUE}=\frac{\left(\text{Yield}\;\text{of}\;\text{fertilized}\;\text{plot}\right)-\left(\text{Yield}\;\text{of}\;\text{control}\;\text{plot}\right)}{\left(\text{Phosphorus}\;\text{applied}\right)}$$

$$\text{AFPUE}=\frac{\left({\text{Phosphorus}\;\text{in}\;\text{fertilized}\;\text{plants}\;\text{ha}}^{-1}\right)-\left({\text{Phosphorus}\;\text{in}\;\text{control}\;\text{plants}\;\text{ha}}^{-1}\right)}{\left(\text{P}\;\text{applied}\right)}$$

$$\text{PIR}=\frac{\text{P}\;\text{economic}\;\text{use}\;\text{efficiency}}{\text{P}\;\text{biological}\;\text{use}\;\text{efficiency}}$$

Statistical analysis was carried out by utilizing the LSD at 5% level of probability [30].

## 3. Results

The data for two years showed non-significant variation hence the pooled data over years has been presented and discussed below.

### 3.1 Nutrient status in soil and in organic sources

The soil of the field study was silt loam having pH 7.2 and 7.1. The pH of poultry manure was 6.82 and 6.55 (Mclean method) in 2011 and 2012, respectively. Soil organic carbon 1.31% and 1.12% (Nelson and Sommers method), total N 0.041% and 0.029% in soil. Olsen’s available P was 6.9 mg/kg and 6.5 mg/kg in soil and Richard’s total extractable K was 177 mg kg^-1^ and 170 mg/kg in soil (Table 1). Total N in poultry manure was 2.21% and 2.33% (Kjeldahl method) in 2011 and 2012, respectively. Total P 1.87% and 1.91% in poultry manure and total extractable K 2.24% and 2.39% during both the years under study, respectively as shown in Fig 1.

**Fig 1:** Percentage of total NPK in poultry manure.

**Table 1:** Physico-chemical analysis of the soil samples from experimental site.

Parameters	2011	2012
Organic matter	1.31%	1.12%
Total N	0.041%	0.029%
Available P	6.9 mg/kg	6.5 mg/kg
Extractable K	177 mg/kg	170 mg/kg
pH	7.3	7.1
Textural class	Silt loam	Silt loam
EC	0.56	0.58

### 3.2 Applied fertilizer phosphorus use efficiency (AFPUE)

The maximum applied fertilizer phosphorus use efficiency (AFPUE) (0.25) was observed in the plots provided with phosphorus SSP+PM@ 60 each kg/ha (Fig 2). While minimum (0.14) AFPUE was observed in P_60SSP_ treatment however plots supplied with P60PM and P90PM also could not reveal significant variation.

**Fig 2:** Effect of various organic and inorganic amendments on applied fertilizer P use efficiency.

### 3.3 Fertilizer phosphorus use efficiency

Significant influence of different P sources on FPUE (Fig 3). The maximum fertilizer use efficiency of phosphorus (23.79) was observed under treatment P_60SSP+60PM_ in which natural and synthetic sources were used in combination at equal doses. It was statistically similar with the P_30SSP+30P,_ P_45SSP+45PM_ and P_60SSP._ Minimum FPUE was observed in the control treatment which was followed by plots supplied with P_60SSP._ The lowest fertilizer phosphorus use efficiency (FPUE) was observed in the P_0_ treatment which was followed by the treatment P_60SSP._

**Fig 3:** Effect of various organic and inorganic P nutrients sources on FPUE* and PIR*.

### 3.4 Phosphorus index ratio (PIR)

Phosphorus index ratio (PIR) illustrated in Fig 3 showed that highest PIR (43.30) was observed in treatment P_60SSP+60PM_ where phosphorus at rate of 60 kg/ha was applied from natural (poultry manure) and synthetic sources of nutrients which was statistically at par with the plot having P_60SSP_ solely. Whereas, the plots P_60PM_ resulted lowest PIR which was followed by plots having P_30SSP + 30PM_ and P_90PM._

### 3.5 Leaf area (cm)

Natural and synthetic sources of P put a substantial influence on leaf area of wheat crop at tillering and heading stages (Fig 4). The maximum leaf area (28.76 cm^2^) at tillering was observed in the treatment P_60SSP+60PM_. While the minimum leaf area (21.44 cm^2^) was observed in P_0_ where, fertilizer was not used. Similarly, the outcomes related to leaf area (cm^2^) at the heading stage demonstrated that the treatment P_120PM_ gave maximum leaf area (31.80 cm^2^).

**Fig 4:** Effect of various organic and inorganic nutrient sources on leaf area of wheat.

### 3.6 Leaf moisture percentage at heading stage

The data related to the percentage leaf moisture content at heading stage are shown in the Fig 5. Usage of SSP and PM in combination @ 45, 60 kg/ha and PM @ 120 gave highest leaf moisture content at the heading stage which was at par with SSP _+_ PM @ 30, PM@ 90, SSP @ 90 and 120 kg/ha. While the minimum (54.3%) moisture content of leaf was recorded in P_0_ treatment, where no fertilizers were used. During this present study, combined application of synthetic and organic sources of fertilizer improves leaf moisture content significantly. Combination of P_60SSP+60PM_ kg/ha showed maximum (81.9%) moisture content of leaf at the heading stage which attributed to better soil moisture conservation by Poultry manure (PM).

**Fig 5:** Effect of various organic and inorganic P nutrient sources on wheat leaf moisture content at heading stage.

### 3.7 PH (cm)

The data regarding PH revealed significant differences among various fertilizer sources treated plots (Table 2). Maximum (56.59 cm) PH was observed in plot having P_90SSP_ which was statistically similar with plots having P_120PM_ and P_60SSP + 60PM._ While minimum PH was recorded in control treatment where not a single source fertilizer was used. In fertilizer treated plot minimum (50.79 cm) PH was recorded in plot having P_30SSP + 30PM._

**Table 2:** Effect of various organic and inorganic P nutrient sources on yield and yield components of wheat.

Treatments	PH (cm)	SL (cm)	Grain (spike^-1^)	TGW (g)	GY (kg/ha)
P_0 (Control)_	49.5 c	8.7 c	43.0 c	29.3 e	1119 f
P_60SSP_	53.6 ab	9.5 bc	47.4 bc	35.3 d	1259 ef
P_90SSP_	56.5 a	10.4 abc	50.0 ab	40.3 abcd	1459 cde
P_120SSP_	54.8 a	11.0 ab	53.2 a	42.0 ab	1773 bc
P_60PM_	54.6 ab	9.6 bc	48.5 ab	37.6 bcd	1277 ef
P_90PM_	53.4 ab	9.8 bc	51.4 ab	40.3 abcd	1428 de
P_120PM_	54.7 a	11.0 ab	50.0 ab	43.3 a	1720 bcd
P_30SSP + 30PM_	50.7 bc	9.1 c	49.4 ab	36.0 cd	1409 de
P_45SSP + 45PM_	54.1 ab	10.9 ab	53.3 a	40.6 abc	1863 b
P_60SSP + 60PM_	54.9 a	11.7 a	53.6 a	43.3 a	2397 a
LSD (*p* ≤ 0.05)	3.88	1.79	5.25	5.26	338.39

Means sharing same letter could not differ significantly at 5% probability level.

(I) Control (P_0_) without application of fertilizer; (II) SSP @ 60kg/ha (P_60SSP_); (III) SSP @ 90kg/ha (P_90SSP_); (IV) SSP @ 120kg/ha (P_120SSP_); (V)PM @60 kg/ha (P_60PM_); (VI) PM @90 kg/ha (P_90PM_); (VII) PM @120 kg/ha (P_120PM_); (VIII) SSP @30 kg/ha + PM @ 30 kg/ha (P_30SSP+30PM_); (IX) SSP @45 kg/ha + PM @45 kg/ha (P_45SSP+45PM_); (X) SSP @60 kg/ha + PM @60 kg/ha (P_60SSP+60PM_).

### 3.8 SL (cm)

Data regarding SL (Table 2) shown that highest (11.79 cm) SL was recorded in SSP @ 60 + PM @ 60 in combination, while minimum (8.78 cm) was recorded in plots which did not receive any P dose from either source.

### 3.9 Grains (spike^-1^)

Maximum number of grains spike^-1^ (53.67) was recorded in plot where integrated application of SSP and PM each @ 60 kg/ha was done. It seems statistically alike to plots P_45SSP+45PM_ and P_120SSP,_ while the minimum grains spike^-1^ were observed in P_0_ (control) treatment where no P was applied reflects the importance of P in wheat grains number.

### 3.10 TGW (g)

Data regarding TGW revealed that heavier 1000-grains were observed in the integrated treatment of P_60SSP + 60PM_ (43.33 g). However, SSP or PM application either at 90 and 120 kg/ha also revealed statistically similar grains on weight basis. While the lighter grains (29.33 g) were observed in P_0_ (control) where fertilizer application was not practiced.

### 3.11 GY (kg/ha)

Results showed maximum GY (2397 kg/ha) in plots where phosphorus was used @ 60 kg/ha from integrated sources (PM and SSP). It was followed by GY 1863 kg/ha by the treatment P_SSP45+PM45_ in which synthetic and organic sources were applied in combination. It could not vary significantly from the wheat plants in plots supplied with P 120 kg/ha from PM. The results show that, there was back to back improvement in the wheat yield of grain with increase in supply of phosphorus by the integrated use of natural (PM) and synthetic (SSP) nutrient sources. Whereas, minimum (1119 kg/ha) GY was observed in the control (P_0_) treatment which was statistically similar with P_60SSP_ and P_60PM_ treated plots. Moreover, P_120SSP_ performed intermediate (1773 kg/ha) which was statistically similar to plots nourished with P_120PM_ showing GY of 1720 kg/ha. It was followed by P_30SSP+30PM_ treated plots (1409 kg/ha) which is statistically different from the P_120SSP_ applied plots.

## 4. Discussion

Presented data showed that maximum AFPUE and PUE was observed plot P_60SSP+60PM_ having natural and synthetic sources at equal doses. The significant difference for AFPUE can be attributed to various responses of different treatments for the uptake of phosphorus in sub-humid environment. The enhancement of AFPUE in P_60SSP+60PM_ could be attributed to the improvement in moisture retention which might have occurred due to better organic matter in soil. Moreover, soil moisture content influence on growth pattern of crop determines the demand of phosphorus for the crop. Application of phosphorus through combined organic and inorganic sources makes the nutrient in that form which was not fixed and was more available owing to improved microbial activity. Roots of crop take up accumulated P in soil as residues from where combined organic and inorganic fertilizers were applied. Combined application of P sources helps them to utilize more nutrients for growth and development [31]. Furthermore, over the period addition of phosphorus and potassium sources in soils, the concentration of these nutrient increases over the time [32, 33]. Application of integrated phosphorus improved nutrient supply, soil health and crop growth. It promoted availability of N and P [34] and improved biomass as well as yield of crop [35]. Grain production per unit use of nutrient (FUE) is an index for effective usage of fertilizers. Better FPUE of treatment P_60SSP+60PM_ could be resulted in improvement in GY yield per unit supply of P nutrients. Moreover, the application of phosphorus @ 60 kg/ha from both natural (PM) and synthetic (SSP) source could be an appropriate prescription that can improve the soil productivity and fertility which leads to maximize the FPUE. Furthermore, improved fertilizer use efficiency of phosphorus in P_60SSP+60PM_ can be attributed in to the increase in the yield of wheat crop per unit use of phosphorus nutrient. FPUE enhanced with appropriate dose application [36].

Phosphorus index ratio presented data showed that substantial increase in the responsiveness of phosphorus for PIR in higher-regimes phosphorus can be attributed to the enhancement in GY of. Probably, wheat plant at high phosphorus doses accumulates and utilizes more phosphorus that increase the economic production leading to higher PIR in the P_60SSP+60PM_ treatment. Phosphorus applied by external sources in appropriate doses can increase yield of crops significantly [37, 38].

In the present study, combined use of natural and synthetic nutrient sources improves the leaf area considerably as compared to P_0_ (control). Results showed that PM sole and integrated form with synthetic P sources significantly improve the growth and yield parameters as compared to control treatment, which revealed the importance of these sources fertilizers to improve productivity. Sole and integrated application of organic and inorganic fertilizer sources could increase the growth parameters [39, 40].

Significant higher leaf moisture percentage in plot where natural and synthetic sources of fertilizer was applied in combination resulted in improved soil physical properties that help to retain the highest leaf-moisture content. Integrated application of synthetic and natural nutrient sources resulted in increased soil moisture conservation, nutrient availability and enhanced biological and economic yield of the crops [41]. Combined use of nutrient sources can help improve soil health by making an improvement in soil physiochemical traits, nutrient cycling, speed up the soil enzyme activities and as well as bioactivities of soils [42] making soluble phosphorus available readily ultimately helping to improve the crop yield. Organic and inorganic P sources have a direct influence on leaf area, moisture contents, growth and development of wheat.

Varying doses of P as sole application either synthetic or natural source could not vary significantly for plant stature as compared to the plots applied with combined application of P from SSP and PM each at 60 kg/ha. The highest plant-height observed can be attributed to the improved vigor of plant, growth of root and the WUE of the crop that could have helped the wheat plant to get maximum height. An improvement in the level of P supply resulted in improvement in the height of the plant [43]. Moreover, application of phosphorus sole or in integration in various ratios can be beneficial, because it helps in mobilizing inherent phosphorus that affect the uptake and usage of phosphorus which helped crop plant in the growth and development [44]. However, reduction in P dose to 30 kg SSP and PM each per hectare reduced the growth of plants reflected in reduced height of wheat plants. The plots not received any P source or dose showed smaller plants. PH is controlled by the environmental conditions [4] as well as genetic properties of crop plant [45].

It was interesting to note that single source of P either SSP or PM each at 60 and 90 kg/ha could not differ significantly from zero applied P source showing similar length of spike. Enhancement in the length of spike could be due to the sufficient availability of moisture and nutrient. Organic sources improve crop productivity by increasing the soil health. So, instead of using sole dose of organic manure and inorganic chemical fertilizers, use of these sources in combination can attain more effective and suitable environment for growth and yield of crop. Application in combined form of fertilizer sources increase the spike-length [46].

Significant higher number grains spike^-1^ in plot where combined dose of organic and SSP were applied at 60 kg ha^-1^. This showed the importance of optimum rate of phosphorus in cereal crop to get potential of grains spike^-1^. Maximum grains s pike^-1^was achieved by the application of higher dose phosphorus [47]. The integrated application of P fertilizer showed higher grains per ear in cereal (maize) field as compared to plot where sole fertilizer treated plots [48].

TGW of wheat plants was high significantly where fertilizers were applied in integrated form. Use of combined 50:50 of P organic and inorganic sources helps to improve grain yield as compared to control treatment [48]. Moreover, optimum dose of phosphorus application helped in achieving maximum 1000 grain weight [47]. This was probably due to improvement in water holding capacity (WHC), uptake and usage of phosphorus increase the rate of photosynthesis and also provide extra opportunity for the transportation of carbohydrates from source to sink (grains). It would have ultimately resulted in increased grain-size and weight of 1000 grains.

Presented data related GY showed that among the sources, SSP fertilized plots @120 kg/ha revealed relatively more GY than the sole PM fertilized plots at the same dose i.e. 120 kg/ha. Application of fertilizer in combined form from organic and inorganic sources resulted to significantly positive influence on crop health as well as on the crop yield. Integrated use of organic manures (irrespective of its kind) and inorganic fertilizer sources enhances the crop yield substantially [49, 50]. The mixture of organic and inorganic sources of fertilizers produces higher yield in wheat crop [51]. Improvement in the size of grains was observed with the combined application of phosphorus fertilizers [52]. GY basically depends on various components particularly moisture, nutrient and 1000-grain weight. So the plot P_SSP60+PM60_ showed maximum yield which could be attributed to the interaction between these yields components. Whereas, the minimum GY observed in P_0_ and P_60SSP_ could be due to reduced P supply which ultimately reflected by the poor plant establishment and low TGW. The results showed the consecutive increase in yield of grains with the increase in the supply of phosphorus in integrated organic and synthetic form. Pre-mixing of SSP with PM enhanced the phosphorus availability in soil and uptake by the plants leading to improvement in GY of crop. Mixing of rock-phosphate with organic manure increase yield of wheat crop [53].

Inorganic fertilizer is also not highly soluble and not easily available to plant roots that’s why phosphorus use efficiency significantly affects the production of wheat crop. Application of synthetic fertilizer increase the PUE that resulted in significantly increase GY [54]. Inorganic P nutrient source always influence GY of wheat because its agronomic nutrient use efficiency is always greater than any other nutrient source [55]. So, significant difference for the GY of wheat can be attributed to higher FPUE of P_120SSP_ treatment in sub-humid environmental conditions. Phosphorus uptake and its usage are controlled by the storage of moisture in the root zone of crop plant [56]. All yield parameters showed significantly different response to different source of P fertilizers which revealed that PM or other synthetic fertilizer to enhance wheat crop growth. Under controlled environment cotton crop growth and development showed similar response when PM was applied [57]. The increase in yield could be attributed to the improvement in phenological parameters which could be attributed to application of organic fertilizers that regulate the growth and physiological processes by regulating the growth chemicals [58]. The organic fertilizers were used in agriculture from ancient days but in recent decades due to low organic matter content and harmful effect of synthetic fertilizer help to understand the importance of sustainable and organic farming [59].

## 5. Conclusion

The present investigations amplified the importance of applying phosphate fertilizers and organic manures in combination for increased wheat grain yields. P_60SSP+60PM_ application makes phosphorus nutrients readily available from the fertilizers used and manure improve the soil properties. Hence it may be concluded that farmers in sub humid areas should apply P in soil in an integrated way with 60 kg/ha each from SSP and PM not only to improve the AFPU, FPUE and PIR but also to obtain higher and sustainable wheat productivity. It will also ensure less reliance on chemical fertilizers and will reduce the subsequent potent risks associated with continuous and heavy use of synthetic fertilizers on aerial and soil environment.

## Supporting information

S1 Data (ZIP)
